This article has been retracted.

# Human Cystathionine-β-Synthase Phosphorylation on Serine227 Modulates Hydrogen Sulfide Production in Human Urothelium

**DOI:** 10.1371/journal.pone.0136859

**Published:** 2015-09-14

**Authors:** Roberta d’Emmanuele di Villa Bianca, Emma Mitidieri, Davide Esposito, Erminia Donnarumm, Annapina Russo, Ferdinando Fusco, Angela Ianaro, Vincenzo Mirone, Giuseppe Cirino, Giulia Russo, Raffaella Sorrentino

**Affiliations:** 1 Department of Pharmacy, University of Naples, Federico II, Via D. Montesano, 49, Naples, Italy; 2 Interdepartmental Centre for Sexual Medicine, University of Naples, Federico II, Via Sergio Pansini 5, Naples, Italy; 3 Department of Molecular Medicine and Medical Biotechnologies, University of Naples Federico II, Via Sergio Pansini 5, Naples, Italy; 4 Department of Neurosciences, Human Reproduction and Odontostomatology, University of Naples, Federico II, Naples, Italy; Emory University, UNITED STATES

## Abstract

Urothelium, the epithelial lining the inner surface of human bladder, plays a key role in bladder physiology and pathology. It responds to chemical, mechanical and thermal stimuli by releasing several factors and mediators. Recently it has been shown that hydrogen sulfide contributes to human bladder homeostasis. Hydrogen sulfide is mainly produced in human bladder by the action of cystathionine-β-synthase. Here, we demonstrate that human cystathionine-β-synthase activity is regulated in a cGMP/PKG-dependent manner through phosphorylation at serine 227. Incubation of human urothelium or T24 cell line with 8-Bromo-cyclic-guanosine monophosphate (8-Br-cGMP) but not dibutyryl-cyclic-adenosine monophosphate (d-cAMP) causes an increase in hydrogen sulfide production. This result is congruous with the finding that PKG is robustly expressed but PKA only weakly present in human urothelium as well as in T24 cells. The cGMP/PKG-dependent phosphorylation elicited by 8-Br-cGMP is selectively reverted by KT5823, a specific PKG inhibitor. Moreover, the silencing of cystathionine-β-synthase in T24 cells leads to a marked decrease in hydrogen sulfide production either in basal condition or following 8-Br-cGMP challenge. In order to identify the phosphorylation site, recombinant mutant proteins of cystathionine-β-synthase in which Ser32, Ser227 or Ser525 was mutated in Ala were generated. The Ser227Ala mutant cystathionine-β-synthase shows a notable reduction in basal biosynthesis of hydrogen sulfide becoming unresponsive to the 8-Br-cGMP challenge. A specific antibody that recognizes the phosphorylated form of cystathionine-β-synthase has been produced and validated by using T24 cells and human urothelium. In conclusion, human cystathionine-β-synthase can be phosphorylated in a PKG-dependent manner at Ser227 leading to an increased catalytic activity.

## Introduction

Hydrogen sulfide (H_2_S) is the third member of the gasotransmitter family that also includes nitric oxide and carbon monoxide [1]. H_2_S is primarily generated by two pyridoxal 5’-phosphate dependent-enzymes, cysthationine-β-synthase (CBS) and cysthationine-γ-lyase (CSE), which employ cysteine and homocysteine as substrates [2–4]. The H_2_S pathway is involved in many physiological and pathological processes in different organs and apparatuses in animal experimental models and in human [5–8]. Recently, a role for the L-cysteine/H_2_S pathway has been proposed in human urogenital tract [9–15]. Within this context, we have previously demonstrated that CBS and CSE are both expressed in the human bladder and that either an H_2_S donor or L-cysteine relaxes human bladder strips. In addition, a prominent role for CBS in the human bladder has also been postulated [10]. It has also been shown that the incubation of full human thickness bladder samples with 8-Bromo-cyclic-guanosine monophosphate (8-Br-cGMP), a stable analogue of cGMP, or dibutyryl-cyclic-adenosine monophosphate (d-cAMP), a stable analogue of cAMP, triggered a significant increase in H_2_S production [10]. These data suggested that the mechanism underlying this effect could involve post-translational modifications. Several enzymes and protein are regulated through post-translational modifications [16–18]. In the current literature a post-translational activation mechanism for CBS has been demonstrated. Indeed, CBS activity is regulated by post-translational modifications through a small ubiquitin-like modifier protein which is correlated with the localization of CBS in the nucleus leading to diminished catalytic activity [19,20]. Post-translational activation of CBS in response to oxidative stress has also been demonstrated [21] but the molecular mechanism(s) and its pertinence to H_2_S generation are not yet known.

In the recent literature, urothelium has been shown to play an important role in the physiopathology of human bladder. The urothelium is the epithelium lining the surface of the urinary bladder, in close contact with the urine. Urothelial cells are specialized to detect both physical and chemical stimuli and their transducer role is enhanced by their close proximity to the urothelium of afferent and efferent autonomic nerves [22]. To date, the functions ascribed to the urothelium include control of permeability, immune responses and cell-cell communication and which seem to play a pivotal role in responding to injuries and infections [23]. Starting from our previous findings, by using human urothelium and T24 human urothelial cell line, herein we define that i) CBS is the main enzyme involved in generating H_2_S ii) the activation of the cGMP/PKG pathway leads to CBS phosphorylation at Ser227, thereby increasing its activity.

## Materials and Methods

### Human tissue

Full thickness bladder dome samples were obtained from patients, aged 61**–**73 years, affected with benign prostatic hyperplasia that underwent open prostatectomy. All patients presented urodynamic obstruction and large prostate volume (>80 ml). We excluded patients affected by bladder stones, urinary infections, detrusor areflexia and a history of urothelial cancer. The experimental protocol was approved by the Local Ethical Committee (School of Medicine and Surgery, University of Naples Federico II, via Pansini, 5; 80131, Naples, Italy). All patients were informed of all procedures and gave their written consent. The samples were cleared of adherent tissue and urothelium and detrusor were carefully dissected, separated and immediately frozen [10].

### RNA purification and quantitative real-time RT-PCR

Total RNA was isolated from human urothelium by use of the TRIzol reagent (Sigma-Aldrich, Milan, Italy), according to the manufacturer’s instructions, followed by spectrophotometric quantization. Final preparation of RNA was considered DNA- and protein-free if the ratio between readings at 260/280 nm was ≥1.7. Isolated mRNA was reverse-transcribed by use of iScript Reverse Transcription Supermix for quantitative real-time RT-PCR (Bio-Rad, Milan, Italy). The quantitative RT-PCR was carried out in CFX384 real-time PCR detection system (Bio-Rad, Milan, Italy) with specific primers by the use of SYBR Green master mix kit (Bio-Rad, Milan, Italy). Samples were amplified simultaneously in triplicate in one-assay run with a non-template control blank for each primer pair to control for contamination or primer-dimers formation, and the ct value for each experimental group was determined. The housekeeping gene (ribosomal protein S16) was used as an internal control to normalize the ct values, using the 2^*-ΔCt*^ formula [24].

### Cell cultures and transfections

Human cell line T24 was cultured in Dulbecco's DMEM with glutamax (Invitrogen, Carlsbad, CA, USA) supplemented with 10% FBS, 2 mM L-glutamine and penicillin–streptomycin 50 U/ml. CBSΔT24 cell line, derived from T24 cell line and stably silenced for CBS, was grown in DMEM supplemented with 10% FBS, 0.1 mM non-essential amino acids (Euroclone), 2 mM L-glutamine, penicillin-streptomycin 50 U/ml and 0.5 μg/ml puromycin (Sigma-Aldrich, Milan, Italy).

Plasmids were transfected in T24 cells and CBSΔT24 cells (2.5 x 10^6^ cells, 60 mm-well plate) by using Lipofectamine 2000 (Invitrogen, Life Technology, Monza, Italy) according to the manufacturer’s instructions [25,26].

### CBS Silencing

To stably silence CBS, T24 cells were seeded the day before transfection in a 60 mm plate. Cells were transfected 24 hours later, with 2 μg of a CBS short hairpin (sh)RNA expressing vector purchased from Santa Cruz Biotechnology (Santa Cruz Biotechnology, Santa Cruz, CA, USA). Transfected cells were selected with 1 μg/ml of puromycin (Sigma-Aldrich) for 7 days and then the CBS depletion was evaluated by western blotting using anti-CBS (Santa Cruz Biotechnology, DBA, Milan, Italy). The cell clone with lowest expression level was selected and used for further experiments. A short hairpin non-silencing construct was used as control.

### Mutagenesis

The WT-CBS cDNA, was cloned into a version of the eukaryotic expression vector pcDNA4/HisMax C (Invitrogen, Life Technology, Monza, Italy) containing the HA epitope. The constructs containing the substitution of single Ser with Ala, i.e. TCC/GCC mutation, were obtained by PCR site-directed mutagenesis using the QuickChange® Lightning Site-Directed Mutagenesis Kit (Agilent Technology, Agilent Technology, Milano, Italy) and the WT-CBS cDNA as template as previously described [27]. All constructs were verified by DNA sequencing.

### Immunoprecipitation and western blotting

T24 cells were starved for 16 hours, incubated with 100 μM of 8-Br-cGMP or d-cAMP (Tocris, UK) for 5, 15 or 30 min and then used for immunoprecipitation assay. Samples were analyzed as previously described [28,29]. The eluted proteins were used in cell free kinase assays, phosphorylation assay in T24 cells and western blotting analysis.

Aliquots of immunocomplexes and protein samples (30μg) were resolved by 12% SDS-PAGE and analyzed as previously described [30,31]. The membranes then were challenged with anti-CBS (Santa Cruz Biotechnology), anti-HA (Santa Cruz Biotechnology), anti-PKA (Cell Signaling Technology), anti-PKG (Cell Signaling Technology), anti-CSE (Novus Biologicals), anti-GADPH (Sigma Aldrich) and anti-phospho-(Ser/Thr) (anti-pS/T; Cell Signaling Technology). The proteins were visualized with enhanced chemiluminescence detection reagent according to the manufacturer's instructions (Pierce, Rockford, IL, USA).

### H_2_S determination

H_2_S production was evaluated according to Stipanuck and Beck [32] with modifications [33,34]. Human urothelium samples were incubated with 8-Br**-**cGMP (100 μM) or d**-**cAMP (100 μM) for 30 min. T24 cells were incubated with 8-Br-cGMP (100 μM) or d**-**cAMP (100 μM) for 5, 15 and 30 min. The incubation time of 15 min was chosen as optimal time and used in all successive experiments in T24 or CBSΔT24 cells. The selective inhibitors of PKG (KT5823, 10 μM, Tocris, UK) or PKA (KT5720, 10 μM, Tocris, UK) were added for 20 min prior to challenge with 8-Br-cGMP or d-cAMP, respectively.

### Cell free phosphorylation assay

CBS-WT and CBS mutant immunocomplexes (HA-CBS WT, HA-CBS S32A, HA-CBS S227A, HA-CBS S525A) were incubated at 30°C in kinase buffer (10 mM MgCl_2_ and 20 mM Tris-HCl, pH 7.4), in presence of PKG (0.05 μM; Sigma-Aldrich, Milan, Italy). Kinase reactions were started by the addition of ATP (50 μM) containing [γ-^32^P] ATP (0.5 μCi) and terminated after 30 min by the addition of 10 μL Laemmli SDS stop solution. Proteins were resolved by 12% SDS-PAGE. Incorporation of ^32^P was visualized by autoradiography.

### Phosphorylation assay in T24 cells

Starved T24 cells were incubated with PKG inhibitor, KT5823 (10 μM), or PKA inhibitor, KT5720 (10 μM) and then treated with 8-Br-cGMP (100 μM) or d-cAMP (100μM) for 5, 15 or 30 min respectively. Next, CBS was specifically immunoprecipitated from protein extracts by using antibodies against the endogenous protein. Immunoprecipitated proteins were separated by SDS–PAGE and the presence of a phosphorylated CBS was evaluated by western blotting using anti-phospho-(Ser/Thr) (Cell Signaling Technology, DBA, Milan, Italy).

Starved T24 cells were transiently transfected with constructs encoding for HA-CBS WT or HA-CBS mutants. After transfection (24h), cells were treated or not with 100 μM of 8-Br-cGMP for 15 min. Samples were collected and WT or mutant proteins were specifically immunoprecipitated by using antibodies against the epitope HA. Immunoprecipitated proteins were separated by SDS–PAGE and the presence of the proteins and their phosphorylated form was investigated by western blotting analysis using anti-phospho-(Ser/Thr).

### Generation and characterization of specific antibody against phosphorylated CBS

Peptide from amininoacids 225–234 (NAS^227^NPLAHYD) containing a single phosphorylated Ser at position 227 has been selected to obtain polyclonal antibodies in rabbits, namely anti-pCBS^Ser227^ (PRIMM srl, Milano, Italy). The purified antibody was used at 1:400 dilutions for western blotting.

### Statistical analysis

All data were calculated and expressed as mean±SE. The results were analyzed using t Student’ test or analysis of variance (ANOVA) followed by Bonferroni, as needed. A p value <0.05 was considered significant.

## Results

### Human tissue

#### CBS and CSE are expressed in human urothelium

Human urothelium expresses both CBS and CSE as demonstrated by western blot (Fig 1A) and quantitative RT-PCR (Fig 1B). Human urothelium homogenates generate detectable amount of H_2_S in basal condition (i.e. in presence of the vehicle). The incubation with L-cysteine (the substrate) significantly increases H_2_S production (p<0.01, Fig 1C).

**Fig 1:** CBS and CSE expression and activity in human urothelium. (A) Both CBS and CSE are expressed in human urothelium as demonstrated by the western blot analysis. Loading in the gel lanes was controlled by detection of GAPDH protein. (B) Human urothelium expresses CBS and CSE mRNA as determined by quantitative RT-PCR analysis. Data were calculated as Δct and expressed as mean±SE of four separate specimens. (C) Human urothelium homogenate incubation with the vehicle (basal) or with L-cysteine (the substrate) generates detectable amount of H_2_S (**p<0.01). (D) The incubation with 8-Br-cGMP significantly increases H_2_S production compared to vehicle (*p<0.05). This effect is abrogated by KT5823, a selective PKG inhibitor (°p<0.05). The stimulation with d**-**cAMP does not affect H_2_S production either in the presence or in the absence of KT5720, a selective PKA inhibitor. H_2_S levels are calculated as nanomoles per milligram of protein/min and expressed as mean±SE of five different specimen.

#### 8-Br-cGMP but not d-cAMP elevates H_2_S levels in human urothelium

8-Br-cGMP, a stable analogue of cGMP, significantly increases H_2_S generation compared to the vehicle (p<0.05, Fig 1D). This effect is reverted by KT5823, a selective inhibitor of PKG (p<0.05, Fig 1D). Conversely, H_2_S levels are not modified by the stimulation with d-cAMP, a stable analogue of cAMP (Fig 1D). PKA blockade, operated by the selective inhibitor, KT5720, does not modify H_2_S production (Fig 1D).

### Human urothelial T24 cell line

#### CBS and CSE are expressed in human urothelial T24 cell line

T24 cell line expresses CBS and CSE (Fig 2A). The incubation of T24 cell homogenate with the vehicle generates detectable amount of H_2_S (Fig 2B). Following incubation with L-cysteine, H_2_S synthesis is significantly increased in comparison to the vehicle (p<0.05, Fig 2B).

**Fig 2:** CBS and CSE expression and activity in human T24 cells. (A) CBS and CSE protein expression in T24 cells and human urothelium tissue. Loading in the gel lanes was controlled by detection of GAPDH protein. (B) T24 cell homogenates generate detectable amount of H_2_S in basal (vehicle) or in stimulated (L**-**cysteine) conditions (*p<0.05 vs vehicle). (C) 8-Br-cGMP incubation causes a significant increase in H_2_S production at 15 or 30 min (°°p<0.001 and °p<0.05 at 15 and 30 min, respectively). Incubation with the PKG inhibitor, KT5823, abrogates the H_2_S production (^###^p<0.001). d**-**cAMP incubation for 5, 15 and 30 min in the presence or in the absence of the PKA inhibitor, KT5720, did not affect H_2_S production. Data are calculated as nanomoles per milligram of protein per min and expressed as mean±SE of six different experiments.

#### 8-Br-cGMP but not d-cAMP elevates H_2_S levels in human urothelial T24 cell line

T24 cells treated with 8-Br-cGMP show a significant increase in H_2_S production as compared to vehicle peaking at 15 min of incubation (p<0.01 and p<0.05, at 15 and 30 min respectively, Fig 2C). The PKG inhibitor, KT5823, abolishes the 8-Br-cGMP-induced effect (p<0.001, Fig 2C). Incubation of T24 cells with either d-cAMP or KT5720, the PKA inhibitor, does not affect H_2_S production (Fig 2C).

#### CBS silencing

T24 cells were depleted of CBS by stably transfecting shRNA specific for CBS. The clone with the lowest expression level e.g. clone F, namely CBSΔT24 cells, was selected for the subsequent experiments (Fig 3A). The H_2_S production observed in T24 cell is virtually abolished in CBSΔT24 cells (p<0.05, Fig 3B).

**Fig 3:** Effect of CBS silencing on H_2_S production in human T24 cells. (A) Generation of CBSΔT24 cells. Five clones resistant to puromycin were screened for CBS expression using western blotting analysis. Clone F was selected for the further experiments. GAPDH was used as a protein loading control. (B) The H_2_S production in CBSΔT24 is markedly lower than in control T24 cells (*p<0.05). Data are calculated as nanomoles per milligram of protein per min and expressed as mean±SE of four different experiments.

#### CBS phosphorylation

T24 cell incubation with 8-Br-cGMP causes an increase of pCBS at the 15 and 30 min time points (p<0.001 and p<0.05 respectively, Fig 4A). The maximum effect is reached after 15 min of incubation with 8-Br-cGMP. Treatment with the PKG inhibitor, KT5823, abolishes CBS phosphorylation induced by 8-Br-cGMP (p<0.001 and p<0.01 at 15 and 30 min respectively, Fig 4A). In contrast, neither d**-**cAMP nor KT5720, the PKA inhibitor, modifies the levels of pCBS (Fig 4B).

**Fig 4:** PKG phosphorylates CBS in T24 cells. (A) CBS is isolated by immunoprecipitation (Ip) from starved T24 cells treated with 8-Br-cGMP or vehicle in the presence or the absence of PKG inhibitor. CBS phosphorylation is evaluated by western blotting assay using anti**-**pS/T. 8**-**Br**-**cGMP treatment causes a time-dependent increase of CBS phosphorylation (*p<0.05, ***p<0.001 vs vehicle; ^###^ p<0.001 vs 5 and 30 min.). PKG inhibition (KT5823) abolishes CBS phosphorylation induced by the 8-Br-cGMP (°°p<0.01 and °°°p<0.001 vs matched time point). (B) CBS is isolated by Ip from starved T24 cells treated with d**-**cAMP or vehicle in the presence or absence of PKA inhibitor. CBS phosphorylation is evaluated by western blotting assay using anti**-**pS/T. The stimulation with d**-**cAMP in the presence or in the absence of PKA inhibitor, KT5720, does not cause changes in phosphorylated CBS level. Data are calculated as % of CBS phosphorylation and expressed as mean ± SE of three separate experiments. (C) Representative protein expression of PKG and PKA in human T24 urothelial cells, urothelium, detrusor muscle and full thickness bladder tissue homogenates. Loading in the gel lanes was controlled by detection of GAPDH protein. PKG is expressed in all samples. PKA is highly expressed in human detrusor and whole bladder but not in T24 cell lines or human urothelium. The blot is representative of three separate experiments.

#### PKG and PKA expression in human urothelial T24 cell, urothelium, detrusor and full thickness bladder

Western blot analysis clearly showed the expression of PKG in all examined samples i.e. human full thickness bladder, urothelium and detrusor, as well as in T24 cells (Fig 4C). Conversely a robust signal for PKA is only detected in the human detrusor muscle and in the full thickness bladder homogenates but not in human urothelial T24 cells or in human urothelium (Fig 4C).

#### PKG-mediated phosphorylation of Ser227 and Ser525 of CBS in cell free assay

Among the sites predicted by computational analysis (GPS 2.1, Group-based Prediction System) [35], we chose those with the highest score e.g. Ser32, Ser227 and Ser525 (Fig 5A). Three constructs encoding for mutated forms of CBS in which Ser32, Ser227 or Ser525, mutated in Ala namely HA-CBS S32A, HA-CBS S227A and HA-CBS S525A, were generated. An high significant reduction of labeling with ^32^P of HA-CBS S227A and HA-CBS S525A but not HA-CBS S32A proteins compared with HA-CBS WT is observed (p<0.001, Fig 5B), as revealed by cell free phosphorylation assay.

**Fig 5:** PKG phosphorylates Ser227 and Ser525 of CBS protein. (A) Schematic representation of CBS protein domains and predicted PKG phosphorylation sites by computational analysis. (B) Proteins from T24 cells transiently transfected with plasmids expressing HA-CBS WT or HA-CBS mutants (HA-CBS S32A, HA-CBS S227A, HA-CBS S525A), are specifically immunoprecipitated with antibodies against the HA epitope. Immunoprecipitates (Ip) are used in a cell free kinase assay and analyzed for incorporation of ^32^P by autoradiography. The same samples are immunoblotted with antibodies versus HA epitope. A significant reduction of labeling with ^32^P in the HA-CBS S227A and HA-CBS S525A proteins compared to HA-CBS WT protein is reported (***p<0.001). Data are calculated as % of CBS phosphorylation and expressed as mean ± SE of three separate experiments. (C) Proteins from T24 cells transiently transfected with plasmids expressing HA-CBS WT or HA-CBS mutants (HA-CBS S32A, HA-CBS S227A HA-CBS S525A), untreated and treated with 8-Br-cGMP are specifically immunoprecipitated with antibodies against the HA epitope. Immunoprecipitates are separated by SDS–PAGE and immunoblotted with anti-pS/T and anti-HA. The activation of PKG by 8-Br-cGMP leads to a highly significant increase of pCBS produced by cells transfected with HA-CBS WT and HA-CBS S32A mutant (***p<0.001 and °°°p<0.001). Levels of pCBS in cells tranfected with HA-CBS S227A and HA CBS-S525A are increased as compared to untreated control (^###^p<0.001 and ^§§§^p<0.001). Levels of pCBS in HA-CBS S227A and HA-CBS S525A are significantly reduced when compared with HA-CBS WT (^çç^p<0.01). Data are expressed as mean ± SE of three different experiments.

#### PKG-mediated phosphorylation of Ser227 and Ser525 of CBS in T24 cells

Activation of PKG by 8-Br-cGMP significantly increases of about 6 fold CBS phosphorylation in T24 cells transfected with HA-CBS WT construct compared with the matched control (p<0.001, Fig 5C). Similarly, phosphorylation of HA-CBS S32A mutant is increased of 5 fold compared with the control (p<0.001, Fig 5C). Of note, the PKG/cGMP-induced phosphorylation of HA-CBS S227A and HA-CBS S525A is significantly and markedly reduced when compared with HA-CBS WT (p<0.01, Fig 5C). The phosphorylation levels of HA**-**CBS S227A and HA**-**CBS S525A mutants are still increased as compared to their matched control (p<0.001, Fig 5C).

#### The mutation of Ser227 impairs PKG-mediated increase of H_2_S production

CBSΔT24 cells were transiently transfected with constructs HA-CBS WT, HA-CBS S227A or HA-CBS S525A mutants and treated with 8-Br-cGMP or vehicle. Ectopic expression of HA-CBS WT or HA-CBS mutants was assayed by western blotting using anti-HA (Fig 6A). Homogenates of HA-CBS WT generate detectable amount of H_2_S; as expected, 8-Br-cGMP causes a significant increase in H_2_S production (p<0.05, Fig 6B). Of note, mutation of Ser227 led to two effects: i) a significant reduction of H_2_S basal production (p<0.05) ii) the abrogation of 8-Br-cGMP-mediated increase in H_2_S production (p<0.001) both compared to WT (Fig 6B). In contrast, mutation of Ser525 does not affect H_2_S production either in basal condition or following 8-Br-cGMP stimulation. In fact, the H_2_S level in these cells is similar to that observed in homogenates from cells transfected with HA-CBS WT.

**Fig 6:** Mutation of Ser 227 impairs PKG-mediated increase of H_2_S production on T24 cells. (A) Western blot analysis of proteins from CBSΔT24 cells transiently transfected with plasmids expressing HA-CBS WT and HA-CBS mutants (HA-CBS S227A, HA-CBS S525A), incubated with 8-Br-cGMP or vehicle for 15 min. Loading in the gel lanes was controlled by detection of GAPDH protein. (B) Production of H_2_S from the same samples. Mutation of Ser227 significantly reduces H_2_S production in basal condition and following incubation with 8-Br-cGMP compared with the paired WT (^#^p<0.05 and ^###^p<0.001). The levels of H_2_S are not affected by the mutation of Ser 525. Indeed, H_2_S levels are similar to those obtained from HA-CBS WT either in basal condition or upon cyclic nucleotide stimulation. 8-Br-cGMP significantly increases H_2_S production in HA-CBS WT and in HA-CBS S525A compared to vehicle (*p<0.05, ^§§§^p<0.001). Data are calculated as nanomoles per milligram of protein per min and expressed as mean±SE of three different experiments.

#### Characterization of the antibody for pCBS at Ser227

A peptide of 10 aminoacids corresponding to residues 225 through 234 of CBS including phosphorylated Ser227 was used to obtain rabbit polyclonal antibody. The phosphopeptide-specific CBS antibody (anti-pCBS^Ser227^) efficiently recognizes CBS protein in human urothelium and in T24 cells (Fig 7A and 7B). Of note, a more robust pCBS specific signal is detected by anti-pCBS^Ser227^ either in human urothelium homogenates (Fig 7A) or in T24 cell lysates treated with 8**-**Br**-**cGMP (Fig 7B and 7C). No difference in signal intensity is appreciable in the same samples incubated with the anti-CBS (Fig 7A and 7B). No other proteins were detected (data not shown).

**Fig 7:** The pCBS^Ser227^ antibody selectively recognizes the CBS phosphorylated form in human urothelium and T24 cells. (A) Expression of CBS phosphorylated form in human urothelium tissue treated or untreated with 8-Br-cGMP for 15 min. Protein extracts are analyzed by immunoblotting using the anti-pCBS^Ser227^ and anti-CBS. Loading in the gel lanes was controlled by detection of GAPDH protein. (B) T24 cells treated or untreated with 8-Br-cGMP for 15 min. Protein extracts are analyzed by immunoblotting using the anti-pCBS^Ser227^ and anti-CBS. Loading in the gel lanes was controlled by detection of GAPDH protein. A more robust pCBS specific signal is detected by anti-pCBS^Ser227^ in lysates from T24 cells treated with 8**-**Br-cGMP. No difference in signal intensity is appreciable in the same samples incubated with the anti**-**CBS. (C) Protein levels are evaluated by densitometric analysis expressed as arbitrary units. (D) Proteins from T24 cells transiently transfected with constructs expressing HA**-**CBS WT or HA**-**CBS S227A and treated with 8-Br-cGMP are specifically immunoprecipitated with antibody against the HA epitope. Immunoprecipitates (Ip) are separated by SDS–PAGE and immunoblotted with anti-pCBS^Ser227^. Note the absence of signal in cells transfected with HA**-**CBS S227A mutant construct.

Specificity of the antibody for the phospho-epitope of CBS was further evaluated in T24 cells transiently transfected with constructs HA-CBS WT or HA-CBS S227A. As shown in Fig 7D, the immunoprecipitated Ser227Ala mutant CBS protein was not recognized by the anti-pCBS^Ser227^. This latter results demonstrates that the presence of phosphorylation at Ser227 site is necessary for the detection of CBS protein by this specific antibody after 8-Br-cGMP challenge.

## Discussion

We have previously shown that incubation of human bladder tissue with the stable analogues of cGMP or cAMP, i.e. 8-Br-cGMP or d-cAMP, leads to increased H_2_S production [10]. It is well established that cGMP and cAMP activate PKG or PKA respectively, which in turn phosphorylate proteins thereby triggering signal transduction [36]. On this basis, we have hypothesized that the effect triggered by 8-Br-cGMP or d-cAMP involves phosphorylation of CBS, leading to an increased catalytic activity.

In order to address this issue, we focused our attention on the urothelium. The choice of the urothelium was driven by the following reasons i) the important role played by the urothelium in bladder pathophysiology ii) the availability of a well characterized human urothelial cell line such as T24 cells.

As a first step we defined whether CBS and/or CSE were involved in driving the H_2_S pathway in human urothelium, comparing this profile with T24 cell line. We found that both human urothelium and T24 cells express CBS and CSE and efficiently convert L-cysteine into H_2_S. Having determined that both enzymes are expressed and are catalytically active, we assessed whether incubation with 8-Br-cGMP or d-cAMP increases H_2_S production. We have demonstrated that 8-Br-cGMP but not d-cAMP causes a significant increase in H_2_S production in both urothelium and T24 cells. The specificity of the effect of 8-Br-cGMP was confirmed by the reversion operated by KT5823, a selective inhibitor of PKG. These results differed from our previous findings where both 8-Br-cGMP and d-cAMP caused an increase in H_2_S production in full human bladder thickness (detrusor muscle *plus* urothelium) [10]. In order to clarify this issue, we investigated the distribution/expression of PKA *versus* PKG in the human bladder. Western blot analysis for PKG and PKA in human urothelium, detrusor muscle, whole bladder and T24 cells clearly show that urothelium as well as T24 cells strongly express PKG as opposite to PKA. This finding explains the lack of the effect of d-cAMP observed in human urothelium and urothelial T24 cells. Having well characterized that human urothelium and T24 cell line act similarly, we have sought to investigate CBS phosphorylation by stimulating T24 cells with 8-Br-cGMP. A clear time-dependent signal of CBS phosphorylation was observed in CBS isolated from T24 cells stimulated with 8-Br-cGMP. The phosphorylation reached the maximum effect at 15 min declining thereafter. CBS phosphorylation in presence of KT5823, a PKG inhibitor, was blunted. In agreement with the finding that both human urothelium and T24 cells have a very low level of PKA, d-cAMP did not trigger CBS phosphorylation. These data strongly indicate that CBS phosphorylation is PKG-dependent. Due to the lack of selective CBS inhibitors [37], in order to further characterize the role of CBS-derived H_2_S in urothelium, we stably silenced CBS in T24 cells. CBS silencing markedly reduces H_2_S production, confirming the major role played by CBS in triggering the H_2_S production. In summary, we have demonstrated that i) T24 cell line mimics human urothelium behaviour ii) cGMP/PKG pathway activation triggers CBS phosphorylation iii) CBS-derived H_2_S is the major source of H_2_S in T24 cells. Through a computational approach, we searched for possible PKG-phosphorylation sites in CBS protein, focusing on the aminoacid sequence known as PKG target consensus, distinct from sequence predicted as PKA-phosphorylation sites. Predicted PKG-phosphorylation sites in CBS were Ser32, Ser227, and Ser525. To experimentally validate these Ser as sites of phosphorylation by PKG, we performed a phosphorylation assay by using proteins from T24 cells transiently transfected with plasmids expressing HA-CBS WT or HA-CBS mutants (HA-CBS S32A, HA-CBS S227A, HA-CBS S525A). The mutation of Ser227 and Ser525 but not Ser32 causes a drastic reduction of CBS phosphorylation. Furthermore, HA-CBS S227A and HA-CBS S525A mutants display a significantly reduced level of phoshorylation when incubated with 8-Br-cGMP. Taken together, these findings show that among predicted PKG-phosphorylation sites, only Ser227 and Ser525 were experimentally validated as sites of phosphorylation by PKG.

To assess the contribution of each phosphorylation sites to the enzyme activity and ultimately to the extent of H_2_S production, we transiently transfected cells lacking CBS (CBSΔT24) with HA-CBS S525A, HA-CBS S227A mutants or HA-CBS WT as a control. Treatment with 8-Br-cGMP did not induce a significant production of H_2_S in the S227A mutant as opposite to S525A mutant. Indeed, the production of H_2_S in S525A mutant is comparable to that induced by 8-Br-cGMP in CBSΔT24 cells transfected with HA-CBS WT. Therefore only the phosphorylation at Ser227 in CBS protein increased H_2_S production.

In order to further confirm our data we generated a specific antibody against the phosphorylated form. The anti-pCBS^Ser227^ recognizes the CBS phosphorylated form in both urothelium and T24 cell line. Challenge of T24 cell with 8-Br-cGMP causes a clear increase in the signal of the anti-pCBS^Ser227^ confirming and validating our previous findings. The specificity of the antibody was also confirmed by the finding that Ser227Ala mutant is not recognized by the anti-pCBS^Ser227^. Thus the phosphorylation at Ser227 site is necessary for recognition of CBS protein by this specific antibody. Interestingly even though Ser525 is also phosphorylated in a PKG-dependent manner, mutation at this residue does not affect H_2_S production. Ser 525 lies within a non-consensus CBS domain that is described as a regulatory region target of the allosteric modulator S-adenosyl methionine. Therefore, it is reasonable to postulate that phosphorylation of Ser 525 may be implicated in the modulation of additional features of CBS protein not as yet determined.

Although additional experiments will be required to understand the control of CBS function by phosphorylation, it is evident that this covalent modification increases CBS activity. Such an outcome may include conformational changes which could allow more efficient binding to substrates or allosteric modulators and regulation of potential binding partners. Herein we demonstrates that in human urothelium as well as in T24 cells CBS-dependent H_2_S generation involves cGMP/PKG mediated phosphorylation of CBS at Ser227.

In the current literature it is widely accepted that the urothelium influences the contractile state of detrusor smooth muscle [23,38]. Indeed, in several studies performed with human or animal tissues, it has been demonstrated that removal of the urothelium increases the contractile response to several different agonists [39,40]. Thus urothelium constitutively releases agents that modulate muscle contractility thereby contributing in a dynamic manner to bladder function homeostasis. Since cGMP/PKG dependent CBS phosphorylation occurs in human urothelium and regulates H_2_S production, we suggest that this mechanism dynamically contributes to bladder homeostasis by controlling detrusor muscle contractility [10].

Finally, the results of this study may not solely be not confined to the bladder since they introduce the concept that changes in H_2_S production driven by CBS, often ascribed in the relevant literature to a generic change in activity, could involve CBS phosphorylation.

## Conclusions

In conclusion, we have demonstrated that i) incubation of T24 cells with 8-Br-cGMP causes a time-dependent increase in CBS phosphorylation reverted by selective inhibition of PKG ii) in T24 cells stably silenced for CBS, H_2_S production is markedly reduced thus supporting a relevant contribution of CBS in triggering H_2_S production in urothelial cells iii) CBS phosphorylation by PKG at Ser227 increases endogenous H_2_S production confirming that, CBS activity can be selectively enhanced in a cGMP/PKG-dependent manner in human urothelium.

Finally, the antibody, directed against the phosphorylated form of CBS, may represent a useful tool to define the pathophysiological role of the H_2_S pathway, in any pathology where CBS is reputed to play a role.
